# Silencing of AKIP1 Suppresses the Proliferation, Migration, and Epithelial-Mesenchymal Transition Process of Glioma Cells by Upregulating DLG2

**DOI:** 10.1155/2022/5648011

**Published:** 2022-01-24

**Authors:** Zhaohui Chen, Haitao Wen, Jinwei Zhang, Xin Zou, Shuihua Wu

**Affiliations:** Department of Neurosurgery, Hunan Children's Hospital, Changsha City, 410000 Hunan Province, China

## Abstract

Gliomas, the most prevalent brain tumors, account for nearly one-third of the all brain and central nervous system (CNS) tumors diagnosed in the USA. The purpose of this study was to discuss the important role of A kinase-interacting protein 1 (AKIP1) in glioma and reveal the potential mechanism. After prediction by CCLE, the expression of AKIP1 was determined by qRT-PCR and western blot. The impacts of AKIP1 knockdown on the proliferation, migration, and invasion were then measured by MTT, colony formation assay, wound healing, and transwell assays. Western blot was used to assess the protein levels of migration and epithelial-mesenchymal transition- (EMT-) related factors. Subsequently, the expression of Disks Large Homolog 2 (DLG2) was predicted by bioinformatics analyses, and the interaction between AKIP1 and DLG2 was confirmed by IP assay, qRT-PCR, and western blot. Finally, DLG2 was further downregulated in glioma cells to detect the association between AKIP1 and DLG2 in the cellular functions of glioma. It was demonstrated that AKIP1 exhibited a high level in glioma cells, and interference of AKIP1 led to reductions in the proliferation, migration, invasion, and EMT of glioma cells. DLG2, which was lowly expressed in glioma cells, demonstrated a negative link to AKIP2. Inhibition of both AKIP2 and DLG2 counteracted the inhibited cellular behaviors on account of AKIP1 interference. To be concluded, this study presented evidence that AKIP1 silencing suppressed the progression of glioma via targeting DLG2, which could provide novel insights to impede the development of glioma.

## 1. Introduction

As the most prevalent brain tumor, glioma accounts for nearly one-third of the all brain and central nervous system (CNS) tumors diagnosed in the USA [1, 2]. Due to the difficulties in recognizing their symptoms as a direct outcome of extensive growth and high invasion of glial cells, the patients generally miss the optimal time for treatment [2]. There are some 18,000 people in the USA diagnosed with malignant glioma and 16,000 dies of these diseases every year [3, 4]. The high incidence and mortality, together with the intricate pathogenesis of glioma, call for deepgoing research on the potential drugs or targets for their treatments.

A kinase-interacting protein 1 (AKIP1), a 23 kDa protein, was originally discovered in breast and prostate cancer cell lines by mRNA screens [5]. Recent report has considered AKIP1 as an independent predictor factor for malignant glioma by virtue of high AKIP1 expression presented in most of glioma patients [6]. CCLE website predicted that the expression of AKIP1 was upregulated in glioma cells. Its expression was reported to be elevated in cervical cancer (CC) cell lines and tissue samples of CC patients [7]. AKIP1 contributed to epithelial mesenchymal transformation (EMT) and metastasis in cervical cancer via PI3K/Akt/IKK*β* signal transduction [7]. Emerging evidence also suggested that the upregulation of AKIP1 in gastric cancer (GC) specimens was implicated in the clinical metastasis and poor prognosis of GC and underlined the significant role of AKIP1 in stimulating the proliferation, migration, and invasion of GC cells by activating Slug-induced EMT [8].

DLGs own a wide range of protein-protein interaction domains, which can regulate cellular functions [9]. It was found by humanbase tool that DLG2 was lowly expressed in patients at the initial stage of glioma, which was associated with poor prognosis. In addition, CGGA database indicated the negative correlation between the expression of AKIP1 and DLG2 in primary and recurrent glioma. The results of CCLE website also showed that the expression of DLG2 was downregulated in glioma. The stimulation of DLG2 expression by circ0106714 could promote Yap phosphorylation, thereby suppressing the progression of colorectal cancer (CRC) [10]. DLG2 was lowly expressed in ovarian cancer (OC), and the inhibition of microRNA-23a inhibited OC cell viability, invasion, and migration by releasing DLG2 [11].

In the present study, we aimed to investigate if AKIP1 was involved in the development of glioma and uncovered the underlying mechanism, which might open up new routes for the treatment of glioma.

## 2. Materials and Methods

### 2.1. Cell Culture

Normal human glial cells HEB and glioma cell lines (U251MG, A172, LN229, and T98G cells) were obtained from the American Type Culture Collection. All cells were maintained in DMEM supplemented with 10% fetal bovine serum (FBS; Gibco) and 1% penicillin-streptomycin (Gibco). A humid incubator at 37°C with 5% CO_2_ was used for cell culture.

### 2.2. Cell Transfection

For cell transfection, T98G cells were digested by trypsin and seeded onto 6-well plates overnight to reach 70% confluence. shRNA-AKIP1-1 and shRNA-AKIP1-2 vectors were used to silence AKIP1 (GeneCopoeia, Inc.), and sh-DLG2-1 and sh-DLG2-2 were used to inhibit DLG2 expression. shRNA-NC served as the corresponding control. Transient transfections were conducted using Lipofectamine 2000 (Life Technologies; Thermo Fisher Scientific, Inc.) as per the manufacturer's recommendations.

### 2.3. Quantitative Reverse Transcription Polymerase Chain Reaction (qRT-PCR)

Total RNA was isolated from transfected T98G cells by Trizol reagent (Thermo Fisher Scientific) based on the manufacturer's instructions. After determining the protein concentration and purity, cDNA was synthesized by a Reverse Transcription Kit (Takara, Dalian, China). SYBR Green real-time PCR Kit (Takara, Dalian, China) was used for the PCR procedure. The primer sequences of AKIP1 were as follows: F, 5′-GAAGGATCCGTCGACATGGAATACTGCCTGGCGGC-3′; R, 5′-GAACTCGAGTCATACGGGGAACACCAAGTCCAC-3′. The primer sequences of DLG2 were as follows: F, GATGACCCTGGCATATTTATTACGA-3′; R, 5′-ACGATAGACCCTGCTTCCTTCA-3′. The primer sequences of GAPDH, which served as an internal reference, were as follows: F, 5′-GAGTCAACGGATTTGGTCGT-3′; R, 5′-TTGATTTTGGAGGGATCTCG-3′. The relative gene expression was analyzed by a comparative 2^-∆∆Ct^ method.

### 2.4. Western Blot

Total protein was extracted from cells using a radioimmunoprecipitation assay (RIPA) kit (R0010, Beijing Solarbio Science & Technology Co. Ltd., Beijing, China). After quantifying total protein concentration by a bicinchoninic acid (BCA) method, proteins were separated by 12% SDS-PAGE and then transferred onto nitrocellulose membranes. Subsequently, the membranes were sealed by 5% nonfat milk for 1 h and then incubated overnight at 4°C by primary antibodies. On the next day, the membranes were incubated with corresponding horseradish peroxidase-conjugated secondary antibody (Santa Cruz, CA, USA) after being washed by PBS for three times. Finally, the protein bands were then measured with an enhanced chemiluminescence detection kit (KeyGen, Nanjing, China).

### 2.5. 3-(4, 5-Dimethylthiazol-2-yl)-2, 5-Diphenyl Tetrazolium Bromide (MTT)

Cells after transfection for 24 h were plated in a 96-well plate containing 200 *μ*l medium at a density of 6000 cells/well. At indicated time, 100 *μ*l culture medium with 20 *μ*l MTT solution was added into each well of the plate, which was then put in an incubator. 4 h later, and formanzan solution was used to dissolve the blue-purple crystals. The OD value was read at the absorbance of 490 nm.

### 2.6. Colony Formation Assay

The transfected cells were collected and plated into a 100 mm dish at a density of 6000 cells/well and cultured for 2 weeks at 37°C. Then, cell colonies were fixed with methanol for 15 min and stained with 0.1% Crystal Violet (Solarbio, Beijing, China) for 0.5 h at room temperature. Lastly, the number of cell colonies was counted, with photographs captured by an optical microscope (Olympus, DX51).

### 2.7. Wound Healing and Transwell

For wound healing, cells were seeded into the upper chamber of a 96-well transwell plate. DMEM medium supplemented with 10% fetal bovine serum (FBS) was added to the lower chamber. After incubation for 48 h at 37°C, vertical linear scratches were created by a sterile 200 *μ*L pipette tip. For transwell, the insert chambers were coated with diluted Matrigel (BD Biosciences), and the other procedures were similar to the cell migration assay. The migrated and invaded cells were stained with 0.1% crystal and counted in three random fields at ×200 magnification.

### 2.8. Immunoprecipitation (IP)

500 *μ*g of total protein was extracted from transfected cells and blocked by 20 *μ*L of protein G agarose beads (Sigma-Aldrich, St. Louis, MO, USA). Then, the supernatant was added with 2 *μ*L of in the appropriate antibody for incubation overnight at 4°C. The antibodies were also purified using protein G agarose beads. Beads that had been washed were resuspended in Laemmli buffer and heated to reach the temperature of 95°C for 10 min. The samples were treated with SDS-PAGE, followed by western blot with the appropriate antibodies.

### 2.9. Statistical Analysis

GraphPad Prism 5.0 was used to implement statistical analyses. The measurement data were expressed as mean ± standard deviation. The student's *t* test was used to compare data between two groups. Multiple comparisons were conducted by one-way analysis of variance (ANOVA). *P* < 0.05 indicated a significant statistical difference.

### 2.10. Bioinformatics Tools

CCLE database (https://sites.broadinstitute.org/ccle) was to test AKIP1 and DLG2 expression in glioma. Humanbase (https://hb.flatironinstitute.org/) and CGCA database (http://www.cgga.org.cn/) were to examine the interplay between AKIP1 and DLG2 in glioma.

## 3. Results

### 3.1. AKIP1 Is Highly Expressed in Glioma Cells

AKIP1, which was predicted by CCLE website to present abnormally high levels in glioma cells, was expected to act as a novel target for the diagnosis and treatment of glioma (Figure 1(a)). To support our hypothesis, qRT-PCR was conducted to verify its levels in various glioma cell lines. As compared to HEB cells that served as control, we found the expression levels of AKIP1 were upregulated to different extents (Figures 1(b) and 1(c)). Among these glioma cells, T98G cells, which exhibited the highest levels of AKIP1, were chosen for the following experiments. In a word, AKIP1 expression was elevated in glioma.

### 3.2. Silencing AKIP1 Suppresses the Proliferation, Migration, and EMT Process of T98G Cells

Subsequently, the effects of AKIP1 on the cellular functions of glioma were investigated. First, we silenced AKIP1 by shRNA, and shRNA-AKIP1-2 was applied for the following assays owing to its relatively better efficiency than shRNA-AKIP1-1 (Figures 2(a) and 2(b)). Results from MTT and colony formation assay in Figures 2(c) and 2(d) exhibited conspicuous lower OD value and fewer colonies in shRNA-AKIP1-2 group than shRNA-NC. The following loss-of-function assays and analyses on related protein expression demonstrated the lower migration and invasion of T98G cells transfected with shRNA-AKIP1-2 (Figures 3(a)–3(c)). On the whole, these results suggested that silencing AKIP1 suppressed the proliferation, migration, and EMT process of T98G cells.

### 3.3. DLG2 Is Decreased in Glioma Cells

To substantiate the prediction that DLG2 expression was decreased in glioma cells from CCLE website, we measured its levels in HEB and T98G cells (Figure 4(a)). It was obvious that compared with control, the mRNA and protein levels of DLG2 were remarkably reduced in T98G cells (Figures 4(a) and 4(c)). These results indicated that DLG2 might be a potential marker for the diagnosis and treatment of glioma, and thus, we next explored its interplay with AKIP1 and attempted to disclose the underlying mechanism.

### 3.4. Silencing AKIP1 Increases DLG2 Expression

Humanbase demonstrated the interplay between AKIP1 and DLG2, and we further employed CGGA database to discover that AKIP1 was in negative association with DLG2 in primary and recurrent glioma (Figures 5(a) and 5(b)). Then, the IP analysis was used to validate the targeted relationship between AKIP1 and DLG2 under physiological conditions, and T98G cells were transiently transfected with a plasmid expressing full-length AKIP1 or DLG2 tagged with DLG2 or AKIP1, respectively. As shown in Figure 5(c), the result demonstrated the strong interaction between them. Intriguingly, when T98G cells were silenced by shRNA-AKIP1-2, DLG2 expression at both mRNA and protein levels was noticeably raised (Figures 5(d) and 5(e)). Taken together, we could easily find that AKIP1 negatively modulated DLG2 expression.

### 3.5. Silencing DLG2 Reverses the Suppressive Effects of AKIP1 Knockdown on T98G Cellular Behaviors

To determine whether AKIP1 exerted effects on the functions of T98G cells via the regulation of DLG2, we then silenced DLG2 by transfecting sh-DLG2-1 and sh-DLG2-2, and sh-DLG2-1 was used for the next experiments owing to its better transfection efficiency. As compared to the shRNA-NC group, the decreased proliferation and fewer formed colonies were observed in the shRNA-AKIP1-2 group, whereas the combined transfection of shRNA-AKIP1-2 and sh-DLG2-1 restored the proliferation and colony formation in T98G cells (Figures 6(a) and 6(b)). In relation to the cell invasion and migration, the attenuated cell invasion and migration abilities due to transfection of shRNA-AKIP1-2 were reverted by sh-DLG2-1, together with elevated MMP2, MMP9, N-cadherin, Vimentin, Snail, and decreased E-cadherin expression (Figures 6(c)–6(g)). Taken together, silencing DLG2 reversed the suppressive effects of AKIP1 knockdown on T98G cellular behaviors.

## 4. Discussion

AKIP1 has been extensively found to serve as an oncogenic regulator that can facilitate growth and metastasis of several tumors via activation of signaling pathways, thereby affecting the progression of various cancers [8, 12]. A retrospective study on the nonsmall cell lung cancer patients indicated the expression of AKIP1 was correlated with tumor characteristics and prognosis of these patients [13]. It also played an essential role in esophageal squamous cell carcinoma and could predict the poor prognosis of breast cancer via Akt/GSK-3*β*/Snail pathway [14, 15]. The latest statistics, which illustrated the negative association of AKIP1 with overall survival of glioma patients, elucidated the potential of AKIP1 to be a novel biomarker for the treatment of glioma [6]. In the present study, overexpressed AKIP1 was also noted in a myriad of glioma cell lines, which was consistent with the public recognition that AKIP1 might exert an oncogenic role in tumor cells. To verify the significance of AKIP1, AKIP1 was silenced in T98G cells, and the proliferation and colony formation of these cells were found to be significantly suppressed. Importantly, further loss-of-function assays demonstrated that the invasion and migration of T98G cells were suppressed by AKIP1 silencing. EMT, which was related to the tumor cell invasiveness and metastasis [16], has been recognized as a critical participant in the remodeling of the glioma microenvironment [17]. Consistent with the previous finding that AKIP1 knockdown enhanced the expression of EMT-related marker E-cadherin in nonsmall-cell lung cancer cells [18], we again confirmed the elevated E-cadherin expression by AKIP1 knockdown in glioma, indicating the involvement of AKIP1 in regulating EMT process for the promotion of glioma.

As the research moved along, DLG2 was recognized to show a binding relationship with AKIP1. Interestingly, albeit not extensive, DLG2 was confirmed to be involved in the mechanism by which multiple tumors could be controlled [19, 20]. The malignant phenotypes of colorectal cancer cells were enhanced by miR-942-5p via targeting DLG2 [10]. Higher expression of DLG2 was related to the survival of neuroblastoma patients, and it was negatively associated with MYCN status and tumor stage [21]. In this study, DLG2 was at a relatively low level in T98G cells. After confirming the binding relationship between AKIP1 and DLG2, it was found that silencing AKIP1 led to the decrease on the mRNA and protein levels of DLG2. Then, we tested if AKIP1 exerted effects on the T98G cell functions to affect the progression of glioma by regulating DLG2. Notably, the inhibitory impacts of AKIP1 insufficiency on the proliferation, migration, invasion, and EMT process of T98G cells were reversed by silencing of DLG2, which indicated that AKIP1 modulated these cell functions so as to affect glioma development by targeting DLG2.

## 5. Conclusion

To conclude, this study presents evidence that AKIP1 silencing suppresses the progression of glioma via targeting DLG2. Importantly, we have noted the significance of AKIP1 in glioma which may be regarded as a potent molecular marker for glioma. This mechanistic study may open up new routes for the application of AKIP1 to glioma therapy. However, our conclusion was only based on in vitro cell model, lacking the validation of in vivo experiments. Future work will be performed to further verify our findings using animal models.

## Figures and Tables

**Figure 1:** AKIP1 is high expressed in glioma cells. (a) The expression of AKIP1 in glioma was analyzed by CCLE database. (b) and (c) The expression of AKIP1 in normal cell HEB and glioma cell lines was detected by western blot (b) and qRT-PCR (c). ^∗∗^*P* < 0.01 and ^∗∗∗^*P* < 0.001 vs. HEB.

**Figure 2:** Silencing AKIP1 suppresses the proliferation of T98G cells. (a) and (b) The protein and mRNA levels of AKIP1 in T98G cells after transfection with corresponding plasmids. (c) The proliferation and (d) colony formation of T98G cells after AKIP1 interference. ^∗^*P* < 0.05 and ^∗∗∗^*P* < 0.001 vs. shRNA-NC.

**Figure 3:** Silencing AKIP1 suppresses the migration, invasion, and EMT process of T98G cells. (a) The migration of T98G cells before and after AKIP1 interference was measured by wound healing assay. (b) The invasion of T98G cells before and after AKIP1 interference was detected by transwell assay. (c) The protein levels of migration- and EMT-related factors in T98G cells before and after AKIP1 interference was detected by western blot. ^∗∗∗^*P* < 0.001 vs. shRNA-NC.

**Figure 4:** DLG2 is decreased in glioma cells. (a) The expression of DLG2 in glioma was analyzed by CCLE database. (b) and (c) The expression of DLG2 in normal cell HEB and glioma cell line T98G was detected by western blot (b) and qRT-PCR (c). ^∗∗^*P* < 0.01 and ^∗∗∗^*P* < 0.001 vs. HEB.

**Figure 5:** Silencing AKIP1 increases DLG2 expression. (a) and (b) The interaction between AKIP1 and DLG2 expression, as demonstrated by Humanbase and CGGA tools. (c) The binding relationship between AKIP1 and DLG2 was confirmed by IP assay. (d) and (e) The protein level (d) and mRNA level (e) of DLG2 in T98G cells before and after AKIP1 interference. ^∗∗∗^*P* < 0.001 vs. shRNA-NC.

**Figure 6:** Silencing DLG2 reverses the suppressive effects of AKIP1 knockdown on T98G cellular malignant behaviors. (a) and (b) The expression of DLG2 in T98G cells after being knocked down. ^∗∗∗^*P* < 0.001 vs. sh-NC. (c) The proliferation, (d) colony formation, (e) and (f) migration, and invasion of T98G cells after AKIP1 and DLG2 interference. (g) The detection of the protein levels of migration- and EMT-related factors in T98G cells after AKIP1 and DLG2 interference by western blot. ^∗∗∗^*P* < 0.001 vs. shRNA-NC; ^##^*P* < 0.01 and ^###^*P* < 0.001 vs. shRNA-AKIP1-2 + sh-NC.

## Data Availability

The data used to support the findings of this study are included within the article.
